# Analysing Hate Speech against Migrants and Women through Tweets Using Ensembled Deep Learning Model

This article has been retracted.

**DOI:** 10.1155/2022/8153791

**Published:** 2022-04-10

**Authors:** Asif Hasan, Tripti Sharma, Azizuddin Khan, Mohammed Hasan Ali Al-Abyadh

**Affiliations:** ^1^Department of Psychology, Aligarh Muslim University, Aligarh 202001, India; ^2^IT Department, Maharaja Surajmal Institute of Technology, New Delhi 110058, India; ^3^Department of Humanities and Social Sciences, Indian Institute of Technology, Bombay Powai, Mumbai 400076, India; ^4^Mental Health-College of Education, Prince Sattam Bin Abdulaziz University, Alkharj, Saudi Arabia; ^5^College of Education, Thamar University, Thamar, Yemen

## Abstract

Twitter's popularity has exploded in the previous few years, making it one of the most widely used social media sites. As a result of this development, the strategies described in this study are now more beneficial. Additionally, there has been an increase in the number of people who express their views in demeaning ways to others. As a result, hate speech has piqued interest in the subject of sentiment analysis, which has developed various algorithms for detecting emotions in social networks using intuitive means. This paper proposes the deep learning model to classify the sentiments in two separate analyses. In the first analysis, the tweets are classified based on the hate speech against the migrants and the women. In the second analysis, the detection is performed using a deep learning model to organise whether the hate speech is performed by a single or a group of users. During the text analysis, word embedding is implemented using the combination of deep learning models such as BiLSTM, CNN, and MLP. These models are integrated with word embedding methods such as inverse glove (global vector), document frequency (TF-IDF), and transformer-based embedding.

## 1. Introduction

Academic literature and political debates continue to focus on the question of free speech. Hate speech is tolerated in some form or another in many countries [1]. While hate speech and hate crimes have traditionally had devastating effects on individuals and communities, hate speech laws are based on substantive equality. Nazi intentions for the annihilation of the Jewish population were followed by public hatred campaigns, which made hate speech an issue in international law following the Second World War [2]. Social media platforms are concerned about inappropriate user-generated content [3]. Hate speech thrives on social media sites like Twitter because of a lack of accountability and lack of control [4]. Even though social media businesses pay people to censor material, the volume of social media posts is too great for humans to keep track of the concerned people. Our goal in this work is to develop a system for automatically detecting hate speech against migrants and woman through tweets using the ensembled deep learning model. In this work, deep learning models have been trained to tackle the challenges provided by the competition for the automatic identification of hate speech against migrants and woman [5]. It is time to stop arguing about the value of women's contributions to society. According to a recently published UNDP report, women's unpaid domestic and care work in Montenegro achieved a predicted value of 122 million euros in the first three months of COVID-19 in 2020 [6]. When it comes to the workplace, over half of all women have experienced a breach of their rights. This is just the beginning; Montenegro has been experiencing a worrying trend of women and girls being subjected to misogynistic attitudes, sexist language, hate speech, bullying, and other forms of intolerance and discrimination. Despite the abundance of evidence that women and girls make significant contributions to society, we have observed a worrying trend of women and girls being subjected to misogynistic attitudes, sexist language, hate speech, bullying, and other forms of intolerance and discrimination. This can be seen in the public realm and media, particularly in social media conversation. When it appears that women are being used as a political pawn by those with divergent political views and ideologies, it is a deeply troubling development that could undo years of steady progress in raising awareness of the importance of safeguarding universal values such as equality and dignity for all. An outbreak of violence against women directly results from COVID-19's pandemic and has already worsened longstanding disparities in the United States.

Deep learning has done a significant work in the area of sentiment analysis. So, this paper has presented the use of deep learning for analysing the hate speech against migrants and the woman. The application of this work is to identify the people or the users who are posting the messages against the woman and the migrants.

The organisation of the paper is as follows: Section 1 describes the introduction of the proposed work. In section 2 literature survey will be discussed, and section 3 covers the methodology section.  Section 4 explains the implementation details with the results, and section 5 defines the conclusion and future work followed by the references in the last section.

## 2. Literature Survey

The second Global Summit on Religion, Peace and Security was conducted from April 29 to May 1, 2019, by the United Nations (UN). The summit's goal was to produce a Plan of Action to oppose hate speech and protect religious minorities and migrants (United Nations, 2019) [7]. Adama Dieng the UN's Speech Adviser for the prevention of Genocide state that “Political opportunism is fueling an increase in the hate speech.” This statement draws the analogies between 1930s Europe and present political climate on the continent [8]. He warned that “big atrocities often begin with little actions and language.” Dieng is worried about the far-right parties' political plans in Europe following the 2015 refugee crisis. Many of these political parties have taken advantage of Europe's migrant policies to set the stage for a broader discussion on migration. As a result, they have successfully entered mainstream politics by appealing to xenophobia and islamophobia. A hostile climate toward migrants has been fostered by their employment of anti-immigrant rhetoric and the dissemination of false information [9]. On the issue of limiting the nationality of migrants' children and their access to public health care, Chilean president Sebastian Piera ran for office. Immigrants have been referred to as “animals” by President Trump [10]. “You see migrants and refugees being insulted and dehumanised daily.” As Dieng pointed out during his remarks at the summit, you hear politicians utilising that segment of the public as a scapegoat. United Nations concerns about hate speech are not new, but the specific extent of antimigrant and antirefugee rhetoric is becoming increasingly crucial. Since the beginning of the year, over one million asylum seekers have arrived in Europe alone, mainly from the war-torn countries of Libya, Iraq, Afghanistan, and Syria. As the number of migrants fleeing conflict has risen, so has the number of attacks, which have grown.

International human rights treaties and soft law instruments are being used to combat hate speech directed towards refugees and migrants. Concerned about this new problem, the UN launched a comprehensive initiative that culminated in July 2018 with UN member states presenting their renewed commitment to human rights and fundamental values of international law in the form of the Global Compact for Migration. This bolstered the UN's agreement to combat xenophobia and other types of prejudice. Even though 152 nations signed the compact, far-right leaders and parties overwhelmingly rejected it, demonstrating the centrality of antimigrant sentiment in their schedule. No international treaty or convention defines hate speech, but it can be found in human rights treaties and soft laws that limit freedom of expression in general. When construed according to international law, domestic laws should give protection against hate speech to refugees, even while hate speech rules are denied domestically. International law provides a clear outline for the concept of prohibited hate speech. To substantiate this claim, this paper will demonstrate that antihate speech legislation complies with international standards on the limits of freedom of expression while also providing sufficient justification for these laws to protect migrants and refugees under international law.

There are many articles based on hate speech detection, but the novelty of this work is to analyse the hate speech against the woman and the migrants using the deep learning model [11].

## 3. Proposed Methodology

Researchers employ neural networks, which are similar to the human brain in that they connect nodes that process and organise information. As a result of the usage of insults, phrases, and other disparaging statements as training data, an intelligent system can “learn” the patterns and structure of language to forecast incoming tweets and identify objectionable ones. Essential pronouns and other factors can fundamentally alter the meaning of a statement in some sentences. “According to a researcher at the University of Jaén, “with our technology and the support of language resources, we can identify expressions associated with hate speech [12].” A study published in ACM Transactions on Internet Technology, entitled 'Detecting Misogyny and Xenophobia in Spanish Tweets Using Language Technologies', describes how the researchers generated four lists of words in Spanish containing offensive and insulting expressions and words against women and migrants. Artificial intelligence uses this information to identify hate speech focused exclusively on these two demographic groups. Researchers at the University of Jaén are constantly adding new lexical resources to this technology, such as dictionaries and word lists, to improve its accuracy and effectiveness.

Previously hate speech was analyzed through machine learning algorithms. Later on, deep learning algorithms are widely used for performing the analysis. This article is also based on a deep learning approach to perform a better analysis in the hate speech analysis. In the first analysis, hate speech is classified against the woman using deep learning models and in the second analysis is to detect whether the hate speech is performed by the individual or the group of people. To perform the implementation, two different datasets are used, i.e., English dataset based on English text, and the next one is Spanish dataset based on Spanish text [13]. The deep learning model is implemented by the convolutional neural networks with different number of max pooling layer, dropout layers, activation function, and many more. The deep learning models are integrated with the word embedding model such as inverse glove (global vector), document frequency (TF-IDF), and transformer-based embedding, the implemented models are the combination of the convolutional neural network, bilong short-term memory, and multilayer perceptron. The description of the following models are as follows:

### 3.1. Datasets

The dataset split into two parts, i.e., training dataset and the testing dataset. In the training dataset, there are 31,963 records, and the testing dataset consists of 17,198 records. These are further split separately into English dataset and the Spanish dataset. The training dataset is used for building the model, and the testing dataset is used for the validation of the model.

### 3.2. Model 1: Global Vector (Glove) with Convolutional Neural Network, Bi-Long Short-Term Memory, and Multilayer Perceptron

In this method, the text dataset based on English and Spanish language is classified using the deep learning model for the analysis of hate speech against woman and migrants. The word embedding is done through the glove model for performing distributed word representation Figure 1 displays the processing of the English and the Spanish text dataset for the hate speech classification with the help of the Glove model and the ensembled deep learning model.

In this model, firstly, the word embedding model is applied, i.e., glove [14]. Glove encodes a corpus into pretrained weights. Next, deep neural networks use this embedding layer as an input layer. Two convolutional layers, two dropout layers, two max-pooling layers, a flatten layer, and a dense layer were all used in the CNN model [15]. A convolution, dropout, and max-pooling layer follow this embedding layer before the flatten and dense layers are applied. A dropout layer followed by a dense layer in subtask is considered the most effective. We utilized an embedding dimension of 300 for each language subtask to minimize losses and get the most accurate results and applied the “Adam” optimizer. The dataset for subtask B was so imbalanced that we used the “ADASYN” oversampling technique to balance the data [16]. Internal activation is based on “ReLU,” and the final output dense layer is on the sigmoid [17].

Two hidden layers of a multilayer perceptron (MLP) integrate the LSTM with the MLP [18]. The LSTM neural network processes word embeddings one at a time while maintaining the order of the words [19]. Hyperbolic tangent activation is used to handle the output of the LSTM neural network. This is a 600-by-600-pixel vector. The MLP network has three layers:

- An input layer with 600 neurons
- A hidden layer with 1,600 neurons and 100 neurons activated by ReLU
- An output layer with the rest of the neurons (a single neuron with sigmoid activation multilayer per function)
- Between each pair of layers, dropout units have been inserted, each with a probability of 0.8%. To avoid overfitting, the dropout units provide a possibility of deletion to each input neuron during training
- All of our models have been built using the Keras library

### 3.3. Model 2: TF-IDF (Term Frequency- Inverse Document Frequency) with Multilayer perceptron, Support Vector Machine, and XGBoost (Extreme Gradient Boosting) Classifier [20]

In this model, the word embedding TF-IDF model is integrated with multilayer perceptron, support vector machine, and XGBoost (extreme gradient boosting) classifier.

(i) TF-IDF (term frequency-inverse document frequency). Documents are distinct from each other based on the terms they use. Classifications are analyzed using the TF-IDF approach to determine the importance of terms. The TF-IDF score of each term or word in the document is used instead of frequency in this method. Similar to the bag of word algorithm, the TF-IDF score of each term replaces the word count.
  (1) $$\begin{array}{c} TF*I\;DF\left(t,d\right)=\;TF_{t,\;d}*\;\frac{\log\;N}{DF_{t}}. \end{array}$$
In the above equation, *TF* represents the term frequency and *I*  *DF* defines the inverse document frequency. *t*, *d*  is showing the number of terms *t* appears in a document *d*. *N* denotes the number of documents.
If you want to calculate the TF-IDF score of an individual phrase inside an entire document, you can do so by multiplying the total number of documents in the document by the frequency of that term (DF) [21].
(ii) Multilayer. Multilayer perceptron is a feedforward artificial neural network (ANN) that includes input and hidden layers and output and feedback layers. Backpropagation is used to update the weights of all nodes in an MLP. During training, nonlinear mapping is learned by utilising nonlinear activation functions and numerous layers. Nonlinear activation is used to generate the label in MLP [22].
(iii) Support vector machine. One of the most common classification and regression algorithms is the Support Vector Machine (SVM), a supervised technique for classification and regression issues. To locate the decision border between two classes, it uses a vector space model that is as far away from the data points as possible, and the support vectors are data points near the hyperplane that divides classes [22, 23].
(iv) XGBoost classifier. In addition to tree-based models, another sort of an ensemble model is a “boosting model.” For example, machine learning ensemble meta-algorithms for minimising bias and variance in supervised learning are known as “boosts.” They are a class of machine learning algorithms that turn weak learners into strong ones. For example, a classifier with a slender correlation with the actual categorization is said to be a weak learner (it can label samples better than random guessing).

### 3.4. Model 3: Transformer Model with Convolutional Neural Network and the Multilayer Perceptron

In this proposed model, the word embedding is done through transformer model; i.e., electra and the classification are performed by using the ensemble convolutional neural network and the multilayer perceptron model.

The electra model is possible to corrupt the input by replacing some tokens with (MASK) and then train a model to recreate them using pretraining approaches such as BERT. To be effective, they typically demand a considerable amount of computing power to perform well in downstream NLP tasks [24]. A more sample-efficient pretraining task termed replacement token detection has been offered as an alternative. By replacing tokens with plausible alternatives from a tiny generator network, the technique corrupts input rather than hiding it. Finally, instead of predicting the original identities of the corrupted tokens, the electra model trains a discriminative model that predicts whether a generator sample replaced each token in the corrupted input. Because this new pretraining job has specified overall input tokens rather than just a limited fraction that was masked away, it is more efficient than MLM, according to a series of rigorous studies.

Given the same model size, data, and computing power, the contextual representations learnt this way beat those trained by BERT. On the GLUE natural language understanding benchmark, an algorithm trained on one GPU for four days outperforms the state-of-the-art GPT (learned using 30 times more CPU) [25]. Regarding performance at scale, the technique is comparable to RoBERT and XLNet while utilising less than a quarter of their computation and surpassing them when using the same amount of computing [26].

## 4. Results and Discussion

To perform the implementation, a python programming language is used. The evaluation parameters used for detecting the models are accuracy, precision, and the F1 score. All the models are implemented separately, and the results are compared. The model implemented using glove and the LSTM has performed better than the other states-of-the-art algorithms. In Tables 1 and 2, comparison results of the proposed method are given. The results shown in Table 1 was generated through the English language dataset, and Table 2 displays the result achieved through the Spanish dataset. All the three above discussed models in section 3 are applied on both datasets, i.e., English and Spanish.

Above Tables 1–4 and Figures 2–5 have shown the comparison of the models based on English and Spanish dataset. The classification is done to perform hate speech classification against the woman and the migrants. The results have shown that the model implemented with the transformer model and the deep learning model has achieved a better accuracy than the other models.

## 5. Conclusions and Future Work

This paper focuses on text categorization in which two datasets are based on English and Spanish languages. These datasets are used for performing the hate speech classification against women and migrants. In the first analysis, three different types of deep learning models based on artificial neural networks are applied to the English dataset for performing the hate speech analysis, and in the second analysis, the same deep learning models are applied to the Spanish dataset. The parameters used for evaluating the model are accuracy, precision, and the F1 score. The model implemented with the transformer word embedding and the hybrid approach of the convolutional neural network and multilayer perceptron has achieved more than 95% accuracy, which is better than the other state-of-the-art algorithms. In the future work, to enhance the classification performance some more algorithms based on convolutional neural networks, capsule networks will be implemented.

## Figures and Tables

**Figure 1:** Glove model with ensemble CNN, BiLSTM, and MLP.

**Figure 2:** Comparison graph of the models based on English dataset for the hate speech classification against a woman.

**Figure 3:** Comparison graph of the models based on Spanish dataset for the hate speech classification against a woman.

**Figure 4:** Graph comparison based on English dataset for the hate speech detection by the individual or group of people.

**Figure 5:** Graph comparison based on Spanish dataset for the hate speech detection by the individual or group of people.

**Table 1:** Model comparison based on English dataset for the hate speech classification against woman.

Model	Accuracy	Precision	*F*1 score
Support vector machine	87.58	86.42	85.43
Multilayer perceptron	88.48	87.38	86.31
Random forest	88.88	87.48	86.36
CNN	93.79	91.9	90.14
Glove-BiLSTM + CNN + MLP	94.81	93.2	92.19
TF-IDF + MLP + SVM + XGB	95.63	94.1	93.2
Transformer-CNN and MLP	95.78	94.6	93.4

**Table 2:** Model comparison based on Spanish dataset for the hate speech classification against woman.

Model	Accuracy	Precision	*F*1 score
Support vector machine	87.51	86.37	85.14
Multilayer perceptron	87.49	86.46	85.43
Random forest	87.83	86.78	85.63
CNN	92.89	91.77	91.01
Glove-BiLSTM + CNN + MLP	93.42	92.74	91.36
TF-IDF + MLP + SVM + XGB	94.65	93.81	92.68
Transformer-CNN and MLP	95.71	94.62	93.52

**Table 3:** Model comparison based on English dataset for the hate speech detection by the individual or group of people.

Model	Accuracy	Precision	*F*1 score
Support vector machine	86.59	85.23	84.76
Multilayer perceptron	87.49	86.23	85.17
Random forest	88.83	87.15	86.33
CNN	94.79	92.23	91.74
Glove-BiLSTM + CNN + MLP	95.61	94.61	93.28
TF-IDF + MLP + SVM + XGB	96.1	95.15	94.17
Transformer-CNN and MLP	96.23	95.23	94.19

**Table 4:** Model comparison based on Spanish dataset for the hate speech detection by the individual or group of people.

Model	Accuracy	Precision	*F*1 score
Support vector machine	87.58	86.47	85.14
Multilayer perceptron	88.48	87.13	86.38
Random forest	88.88	87.52	86.46
CNN	93.79	92.16	91.53
Glove-BiLSTM + CNN + MLP	94.23	93.49	92.43
TF-IDF + MLP + SVM + XGB	95.12	94.76	93.71
Transformer-CNN and MLP	95.63	94.39	93.82

## Data Availability

Dataset has been downloaded from the https://www.kaggle.com/dv1453/twitter-sentiment-analysis-analytics-vidya?select=test_tweets_anuFYb8.csv, and some more content is added in the dataset through Extracting Tweets from Twitter using tweepy library.
